# Efficacy and Safety of Convalescence Plasma Therapy in COVID-19 Patients: A Systematic Review and Meta-Analysis

**DOI:** 10.1155/2022/7670817

**Published:** 2022-10-07

**Authors:** Rongjuan Dai, Minjie Hu, Haibo Tang, Zhongtian Peng, Cai Yan

**Affiliations:** ^1^The First Affiliated Hospital, Department of Infectious Diseases, Hengyang Medical School, University of South China, Hengyang 421001, Hunan, China; ^2^The First Affiliated Hospital, Department of Cardiothoracic Surgery, Hengyang Medical School, University of South China, Hengyang 421001, Hunan, China

## Abstract

**Background:**

The coronavirus disease 2019 (COVID-19) has outbroken into a global pandemic. The death rate for hospital patients varied between 11% and 15%. Although COVID-19 is extremely contagious and has a high fatality rate, the amount of knowledge available in the published literature and public sources is rapidly growing. The efficacy of convalescent plasma (CP) therapy for COVID-19 is controversial.

**Objective:**

This meta-analysis was designed to assess the efficacy of CP therapy for COVID-19 through a literature survey.

**Methods:**

Until August 30, 2021, a literature search was undertaken in Pubmed, Embase, Web of Science, Cochrane Central Register of Controlling Trials (Central), and China National Knowledge Infrastructure databases. The Risk Ratio (RR) and 95% confidence intervals (CIs) were pooled using a fixed or random effect model in dichotomous data. Mean difference (MD) and 95% confidence intervals (CIs) were pooled using a fixed or random effect model in continuous data. Studies with missing or unsuitable data were presented descriptively in the outcomes.

**Results:**

In total, thirteen randomized controlled trials (RCTs) were selected for the present meta-analysis, which included a total of 13232 participants. Our results revealed that the CP group has lower mortality compared to the control group, and there was a statistically significant difference (RR: 0.70, 95% CI: 0.55, 0.89, *Z* = 2.92, *P* = 0.004 < 0.01); other secondary outcomes such as the shortness of breath symptom improved significantly in CP group (RR:1.48, 95% CI: 1.13, 1.93, *Z* = 2.85, *P* = 0.004 < 0.01), as well as Interleukin-6 (IL-6) (MD: −4.46, 95% CI: −8.28, −0.63, *Z* = 2.28, *P* = 0.02 < 0.05) and Ferritin (MD: −447.68, 95% CI: −501.75, −393.6, *Z* = 16.23, *P* < 0.00001) are reduced significantly in CP group. However, there was no statistically significant change in the ventilator withdrawal rate, imaging results improvement, or days to hospital discharge. There was also no substantial difference in viral nucleic acid negative conversion rate and neutralizing antibody-positive conversion rate, as well as the incidence of adverse reactions.

**Conclusions:**

The safety and potential efficacy of convalescent plasma therapy offer a promising treatment strategy for COVID-19. CP therapy can reduce mortality and improve breath and inflammatory cytokines IL-6 and Ferritin in COVID-19 with no significant increase in adverse reactions. However, it does not affect improving virology indicators. In summary, more high-quality clinical trials are needed to verify the conclusion of the present study.

## 1. Introduction

In December 2019, several patients in Wuhan, Hubei Province of China, were diagnosed with pneumonia of unknown etiology [1]. In January 2020, the Chinese Center for Disease Control and Prevention (CDC) confirmed a patient's throat swab sample as the source of Novel Coronavirus, which the World Health Organization (WHO) subsequently designated as coronavirus disease 2019 (COVID-19). Novel coronavirus pneumonia, also known as COVID-19, is a viral respiratory syndrome caused by SARS-CoV-2 (Severe Acute Respiratory Syndrome Coronavirus Type 2) [2]. On March 11, 2020, the WHO announced that the spread of coronavirus disease in 2019 will pose persistent and significant difficulties to the global community.

SARS-CoV-2 infection not only influenced human beings' daily activities [3] but also damaged organs. Evidence showed that SARS-CoV-2 directly or indirectly activates inflammasomes. The inflammatory cytokines lead to pyroptosis, an inflammatory form of cell death, amplify the destructive tissue damage via endothelial dysfunction and vasodilation, promoting endothelins and then resulting in tissue damage and developing into a variety of clinical symptoms [4]. In extreme circumstances, this inflammatory response can cause numerous organ failures [5]. When faced with this scenario, we must act swiftly to present therapeutic choices. Despite advances in vaccination and drug research, including nanotechnology-based drug [6]and natural bioactive molecules [7, 8], unfortunately, due to the genetic diversity and rapid evolution of this novel coronavirus, there is still no special effective treatment has been found to contain the disease [9–11]. General supportive care for novel coronavirus pneumonia is currently the only choice [12]. As is known to all, passive immunity has played an important role in treating infectious diseases [13]. The most recent anti-SARS-CoV-2 treatment, AZD7442, was developed using antibodies isolated from B cells collected from SARS-CoV-2 infected patients and is effective. Still, it is so expensive that is difficult to become widely used [14].

Convalescent plasma (CP) therapy is a form of passive immunity in which antibody-rich blood is collected from recovered patients and infused into other patients after treatment. CP therapy was evaluated in treating Severe Acute Respiratory Syndrome (SARS) in 2003 [15], followed by the Middle East respiratory syndrome (MERS) epidemic [16] and the Ebola epidemic [17]. There is evidence that receptor binding domain-specific antibodies with strong anti-viral activity have been found in the convalescent plasma survivors of novel coronavirus pneumonia [18]. In the first few days of the novel coronavirus pneumonia pandemic, due to a seemingly reasonable mechanism of action, CP generated great enthusiasm [19].

Recently, reports of improvement results of novel coronavirus pneumonia after CP transfusion have been recorded in randomized clinical trials [20, 21]. However, there is still disagreement over the effectiveness of convalescent plasma therapy for COVID-19. Data on the performance of CP in the treatment of novel coronavirus pneumonia that has been reported will be summarized through this systematic review and meta-analysis.

## 2. Methods

### 2.1. Inclusion and Exclusion Criteria

Studies eligible for inclusion must meet the following criteria [22]: (1) include patients diagnosed with COVID-19; (2) only select the published type of RCT; (3) choose CP therapy for intervention; (4) compare the CP with the standard of care (intervention arm) with a standard of care alone (control arm); (5) complete data on intervention group and control group. We excluded review articles, case reports, and case series.

### 2.2. Search Strategy and Study Selection

The reporting of our systematic review and meta-analysis follows the criteria for recommended reporting items for systematic reviews and meta-analyses (PRISMA) [23]. We searched for COVID-19 and COVID-19 serotherapy in Pubmed, Embase, Web of Science, Cochrane Central Register of Controlling Trials (Central), and China National Knowledge Infrastructure through August 30, 2021. Studies that are already included can be used in various languages. The two authors independently reviewed the abstracts of all publications to determine their eligibility.

### 2.3. Study Outcome Measures

The primary outcome is mortality, which refers to all causes of mortality from the time of randomization to the clinical observation endpoint. Secondary outcomes are: (1) clinical improvement rate includes the rate of improvement of shortness of breath, the rate of taking off the ventilator, the improvement of imaging results, the degree of improvement in inflammatory indicators, the degree of improvement of other indicators; (2) incidence of adverse reactions were defined as causes discomfort or pain after treatment that is incompatible with the purpose of treatment; (3) days to hospital discharge that was defined as the number of days from admission to discharge; (4) The improvement rate of virology indicators was analyzed from viral nucleic acid negative conversion rate and neutralizing antibody-positive conversion rate. The viral nucleic acid negative conversion rate was defined as PCR results of COVID-19 virus nucleic acid turned negative. The neutralizing antibody-positive conversion rate was defined as the patient's neutralizing antibodies to COVID-19 changed from negative to positive.

### 2.4. Literature Screening and Data Extraction

Endnote X9 software was used to manage the articles we obtained. Two independent investigators selected titles and abstracts that were no longer supported by literature searches for inclusion in the study. Further analysis of the full text was carried out after reading the abstract and finding that it does not explicitly meet the inclusion criteria. A third investigator was responsible for discussing and resolving any disagreement regarding a study selection. If there was a disagreement in the data extraction, which was done independently by the two reviewers using a standard data extraction form, the arbitrator reviewed and evaluated it [22]. First author, country, year of publication, design, sample size, treatment of patients in the group (CP group and control group), CP dose, outcomes. The information mentioned above belongs to the main components of the extracted data.

### 2.5. Risk of Bias Assessment

According to the Cochrane Handbook for Systematic Reviews of Interventions, the risk of bias assessment was carried out [22]. The methodological quality of eligible RCTs was evaluated independently through the Cochrane Handbook for Systematic Reviews of Interventions. Specifically, it includes (1) Selection bias: which describes in detail the method for generating randomly assigned sequences; (2) The implementation of bias: concealment of allocation; (3) Measurement bias: blinding of participants, personnel, and outcome assessors; (4) Follow-up of bias: incomplete data on outcome; (5) Reporting bias: selectively reporting favorable results and hiding unfavorable ones; (6) Other biases: conflict of interest, insufficient sample size, unbalanced baseline. Each entry was assessed as “low risk,” “unclear risk,” or “high risk” regarding this statement.

### 2.6. Statistical Analysis

The statistical evaluation was carried out using Stata 16 and RevMan 5.4. If there were two or more homogenous studies available, we used aggregated data [22]. We calculated the risk ratio (RR), 95% confidence intervals (CI), and *P* values for dichotomous outcomes. The mean difference (MD), 95% CI, and *P* values were applied for continuous variables. The *I*^2^ statistics were used to evaluate the study heterogeneity. When *P* ≥ 0.1 and *I*^2^ < 50% indicates no heterogeneity present, *P* < 0.1 or *I*^2^ ≥ 50% indicates heterogeneity [22]. If heterogeneity exists, sensitivity analysis was used to find the source of heterogeneity. Finally, Funnel plots were used for assessing publication bias, with *P* < 0.05 considered significant for publication bias assessment [22].

## 3. Results

### 3.1. Literature Selection

Forty-six articles were retrieved and examined after the abstracts and titles of 760 records obtained by the search method were scrutinized. 13 RCTs satisfied the requirements for inclusion. At the same time, the remaining publications were disqualified for lacking control groups, being nonrandomized controlled trials, or being retrospective research. The process of screening the articles is depicted in Figure 1 flowchart.

### 3.2. Characteristics of the Included Studies

Table 1 demonstrates the characteristics of the 13 randomized clinical trials that were considered [24–36]. There were 254 study centers and 13232 individuals, and all had confirmed COVID-19 diagnoses. The language of all papers was English and from June 2020 to August 2021 were the publication years.

### 3.3. Risk of Bias within Studies

The bias assessment and summary risk are shown in Figures 2 and 3, respectively. The 13 randomized controlled trials included in this study all adopted appropriate methods for randomization, among which 11 used computer-generated randomization [24, 26–35] and 1 randomized controlled trial selected the same paper cards and numbered them sequentially [36]. The last randomized controlled trial was simple randomization of sequentially numbered opaque sealed envelopes [25]. In terms of ensuring the concealment of the distribution scheme, a total of 10 studies described how to ensure the concealment of the distribution scheme, which was judged to be low risk [24, 25, 27, 29–35]. The remaining 3 studies lacked any description of the allocation hiding method, which was considered to have an unclear bias risk [26, 28, 36]. The following methods respectively concealed the 10 studies: (1) Randomized block design treatment assignment [24]; (2) the study personnel received a sealed opaque envelope with an assignment to intervention or control group [25]; (3) Use SAS software and interactive randomization tools in REDCap (Research Electronic Data Capture) [27, 34]; (4) Random assignment was unstratified and done by local clinical or research staff using a web-based interface with allocation concealment [29]; (5) Treatment assignments were generated using randomly permuted blocks [30, 31, 33]; (6) The individual recruiting the patient (senior physician responsible for therapeutic intervention) contacted the center by phone after the patient is enrolled. The respondent in the center was the second researcher, who had designed a table of the 6-item randomized block by computer and added concealment codes without knowing the patient's medical conditions [32]; (7) A central trail coordination team member provided one RCT with random sequences. The nine RCTs were judged to have high risks of performance deviation and detection deviation [25, 26, 28–30, 32, 33, 35, 36]. All 13 RCTs were judged to be low risk in terms of data integrity and selective reporting of results. None of the 13 randomized controlled trials involved conflicts of interest, small sample sizes, or unbalanced baselines.

### 3.4. Analysis of Results

#### 3.4.1. Mortality

At the time of meta-analysis, twelve studies [25–36] compared mortality changes of randomized controlled participants. Those studies in the cluster were tested for heterogeneity (when *I*^2^ = 41.5% < 50%, *Q* test *P*=0.065 < 0.1), indicating that the heterogeneity among the studies is statistically significant. Therefore, heterogeneity needs to be searched. The sensitivity analysis of the 12 studies found that Peter et al. [29] greatly influenced heterogeneity. After removing this study, the effect variables combined in the meta-analysis were large, as shown in Figure 4. Therefore, after removing the study, the results of heterogeneity again showed that there was no heterogeneity in the remaining 11 studies (when *I*^2^ = 11% < 50%, *Q* test *P*=0.34 > 0.1, Figure 5), and this meta-analysis was performed using a fixed effect model after exclusion. There was a significant statistical difference (RR: 0.70, 95% CI: 0.55, 0.89, *Z* = 2.92, *P*=0.004 < 0.01, Figure 5). According to this, patients who underwent convalescent plasma therapy had a 0.70-times higher mortality risk than those who received standard care or a placebo. This shows that patients with COVID-19 may live longer while receiving convalescent plasma treatment.

#### 3.4.2. Clinical Improvement Rate

*(1) The Rate of Improvement of Shortness of Breath*. Three RCTs reported the rate of improvement of shortness of breath [24, 35, 36], and there was substantial statistical heterogeneity among these studies (when *I*^2^ = 84.9% > 50%, *Q* test *P*=0.001 < 0.1). The sensitivity analysis of the three studies found that the study of Agarwal et al. [35] had a great influence on heterogeneity, as shown in Figure 6. Therefore, after removing this study, the results of heterogeneity again showed that there was no heterogeneity in the remaining two studies (when *I*^2^ = 0% < 50%, *Q* test *P*=0.45 > 0.1, Figure 7). There was a statistically significant difference between studies (RR:1.48, 95% CI: 1.13, 1.93, *Z* = 2.85, *P*=0.004 < 0.01, Figure 7). This demonstrated that patients undergoing convalescent plasma therapy had a breath rate improvement rate that was 1.48 times higher than patients receiving standard care or a placebo. It has been suggested that convalescent plasma therapy can help COVID-19 patients with breathlessness.

*(2) The Rate of Taking Off the Ventilator*. The rate of taking off the ventilator was evaluated in six RCTs [25, 28, 29, 32, 33, 35]. No heterogeneity was observed among these studies (when *I*^2^ = 46% < 50%, *Q* test *P*=0.1, Figure 8). The fixed effects model was performed directly, revealing no significant difference (RR: 0.99, 95%CI: 0.90, 1.08, *Z* = 0.28, *P*=0.78 > 0.05, Figure 8). Therefore, it can be concluded that convalescent plasma therapy is not effective in improving the rate of taking off the ventilator.

*(3) The Improvement of Imaging Results*. The imaging results were improved in two RCTs [24, 25], and there was a large statistical heterogeneity among the studies (when *I*^2^ = 78% > 50%, *Q* test *P*=0.03 < 0.1, Figure 9). The random model was used for these analyses. The results showed that there was no significant difference. It is suggested that convalescent plasma therapy is ineffective in improving imaging results (RR:1.77, 95% CI: 0.21, 14.73, *Z* = 0.53, *P*=0.60 > 0.05, Figure 9).

*(4) The Degree of Improvement in Inflammatory Indicators*.

1. CRP: The improvement in inflammatory indicators was examined in four RCTs [24, 25, 28, 32]. A strong heterogeneity among studies (when *I*^2^ = 98% > 50%, *Q* test *P* < 0.1) was observed. As shown in Figure 10, sensitivity analysis cannot identify the study that significantly impacted heterogeneity. Employing the random effect model as a result. The CRP did not differ significantly. According to certain reports, convalescent plasma treatment cannot lower CRP (MD: −40.16, 95% CI: −92.20, 11.89, *Z* = 1.51, *P*=0.13 > 0.05, Figure 11).
2. Ferritin: We analyzed Ferritin in four RCTs [24, 25, 28, 34]. There is strong heterogeneity among studies (when *I*^2^ = 96% > 50%, *Q* test *P* < 0.1). The sensitivity analysis of the four studies revealed that the study of Simonovich et al. [34] had reported a great influence on heterogeneity, as shown in Figure 12. After removing the study, the results of heterogeneity again showed that there was no heterogeneity in the remaining 3 studies (when *I*^2^ = 47% < 50%, *Q* test *P*=0.15 > 0.1, Figure 13), using a fixed effect model after exclusion. With a difference of 447.68 between the two groups, there was a significant difference, revealing that patients who received convalescent plasma therapy had lower Ferritin than those who received standard of care or a placebo, implying that convalescent plasma therapy is effective in lowering Ferritin in COVID-19 patients (MD: −447.68, 95% CI: −501.75, −393.6, *Z* = 16.23, *P* < 0.00001, Figure 13).
3. IL-6: IL-6 levels were examined in two RCTs [28, 32], with no heterogeneity among these studies (when *I*^2^ = 22% < 50%, *Q* test *P*=0.26 > 0.1, Figure 14). There was a significant difference in IL-6 between the CP group and the control group after the fixed model was used. This suggested that participants undergoing convalescent plasma therapy had lower IL-6 levels than those receiving conventional care or placebo, with a 4.46-point difference between the two groups. Convalescent plasma treatment may be useful in lowering IL-6 levels in COVID-19 patients (MD: −4.46, 95% CI: −8.28, −0.63, *Z* = 2.28, *P*=0.02 < 0.05, Figure 14)

*(5) The Degree of Improvement of Other Indicators*

1. Lymphocyte: The level of lymphocytes was assessed in four RCTs [24, 25, 28, 32], and no significant heterogeneity among these studies was found (when *I*^2^ = 22% < 50%, *Q* test *P*=0.28 > 0.1, Figure 15). There was no significant difference in lymphocytes. It is suggested that convalescent plasma therapy is not effective in lymphocyte (MD: 0, 95% CI: −0.03, 0.03, *Z* = 0.14, *P*=0.89 > 0.05, Figure 15).
2. D-Dimer: The D-Dimer was evaluated in two RCTs [24, 34], and there was a large statistical heterogeneity among these studies (when *I*^2^ = 98% > 50%, *Q* test *P* < 0.1, Figure 16), hence the random effects model was used. The findings revealed no significant difference between the CP and control groups. It has been hypothesized that convalescent plasma treatment is ineffective in D-Dimer patients (MD: −518.45, 95% CI: −1754.24, 717.34, *Z* = 0.82, *P*=0.41 > 0.05, Figure 16).

#### 3.4.3. Incidence of Adverse Reactions

Incidence of adverse reactions was tested in thirteen RCTs [24–36], revealing a significant statistical heterogeneity among studies (when *I*^2^ = 57% > 50%, *Q* test *P*=0.02 < 0.1). The sensitivity analysis of the 13 articles revealed that the studies of Peter et al. [29] and O'Donnell et al. [33] had reported a great influence on heterogeneity, as shown in Figure 17. Therefore, after removing the two studies, there was no heterogeneity in the remaining 11 studies (when *I*^2^ = 19% < 50%, *Q* test *P*=0.28 > 0.1, Figure 18). The results revealed that there was no significant difference between the CP and control groups. This indicates that convalescent plasma therapy does not affect the occurrence of adverse events in COVID-19 patients (RR:1.55, 95% CI: 1.00, 2.39, *Z* = 1.95, *P*=0.051 > 0.05, Figure 18).

#### 3.4.4. Days to Hospital Discharge

Six RCTs [25, 26, 28, 32, 33, 35] reported the days to hospital discharge. Heterogeneity test results indicate heterogeneity among these studies (when *I*^2^ = 89% > 50%, *Q* test *P* < 0.01). Sensitivity analysis was performed on these 6 studies to find heterogeneous causes, and we cannot find the study that greatly influenced heterogeneity, as shown in Figure 19. A random effect model was used for the meta-analysis, and there was no discernible difference. It is suggested that convalescent plasma therapy is ineffective in shortening the days to hospital discharge (MD: −0.06, 95% CI: −2.78, 2.65, *Z* = 0.04, *P*=0.96 > 0.05, Figure 20).

#### 3.4.5. The Improvement Rate of Virology Indicators

*(1) Viral Nucleic Acid Negative Conversion Rate*. Viral nucleic acid negative conversion rate analysis was reported in four RCTs [24, 28, 30, 35] with significant heterogeneity (when *I*^2^ = 54% > 50%, *Q* test *P*=0.114 > 0.1). The sensitivity analysis of the four studies found that one study [35] had reported a significant influence on heterogeneity, as shown in Figure 21. Therefore, after removing the study, the results of heterogeneity again showed that there was no heterogeneity in the remaining three studies (when *I*^2^ = 0% < 50%, *Q* test *P*=0.05 > 0.1, Figure 22). There was no significant difference in viral nucleic acid negative conversion rate. It is suggested that convalescent plasma therapy is ineffective in viral nucleic acid negative conversion rate (RR: 0.59, 95% CI: 0.32, 1.11, *Z* = 1.63, *P*=0.1 > 0.05, Figure 22).

*(2) Neutralizing Antibody-Positive Conversion Rate*. Neutralizing antibody-positive conversion rate was tested in two RCTs [24, 36], and there was a statistical heterogeneity among the studies (when *I*^2^ = 53% > 50%, *Q* test *P*=0.15 > 0.1, Figure 22), so the random effects model was used. The findings revealed no discernible difference between the control group and the patients getting CP therapy. It is hypothesized that convalescent plasma therapy is ineffective in reducing positive antibody conversion rate (RR:6.33, 95% CI: 1.00, 40.1, *Z* = 1.96, *P*=0.05, Figure 22).

#### 3.4.6. Publication Bias Detection

Then, we identify publication bias for the meta-analyses of mortality and the incidence of adverse effects. The mortality results indicate that there was no publication bias (*P* > 0.05) (Figure 23(a)); however, the publication bias identification of adverse reaction incidence implies that there may be publication bias (*P* < 0.05) (Figure 23(b)). Other outcomes of the publication bias did not occur since the number of included publications was less than 10.

## 4. Discussion

Measures to treat infectious diseases with CP therapy have been developed for a long time. Many diseases, such as SARS [15], and the 2009 influenza A (H1N1) pandemic, have been well documented [37]. Previous studies have shown that the short-term mortality rate can be reduced in COVID-19 patients treated with severe respiratory failure with CP therapy [38]. However, it was recently reported in severe COVID-19 that CP therapy has nothing to do with clinical benefits [39]. The effectiveness of CP in the treatment of COVID-19 is controversial. In terms of size and test indicator coverage, the current meta-analysis is the largest RCT study meta-analyzed on the COVID-19 fatality research. These results provide evidence that CP therapy can reduce motility and, to some extent, improve clinical presentation. In this meta-analysis, 13 RCTs were included with a systematic review and meta-analysis to evaluate CP therapy in treating the novel coronavirus pneumonia. The analysis showed that most patients tolerated CP transfusions well and that CP therapy was safe. The CP group had a considerably reduced death risk than the control group. The CP group considerably decreased inflammatory indicators, including IL-6 and Ferritin. In terms of clinical manifestation, there was a clear improvement in the CP group's shortness of breath. These findings support the effectiveness of convalescent plasma as a COVID-19 treatment strategy.

As shown in our analysis, CP treatment could not increase SARS-CoV-2 clearance ability in COVID-19 patients but have benefits in reducing mortality. Reductions in inflammatory indicators such as chemokines, cytokines, IL-6, and ferritin protein may be linked to the process through which CP therapy lowers mortality. The neutrophils and lymphocytes in this investigation did not significantly differ between the two groups. CP therapy, however, resulted in significantly lower plasma levels of inflammatory cytokines than the control group. Those results indicated that the possible mechanism of CP treatment might be reducing inflammatory markers, improving gas exchange, reducing oxygen requirements, and improving shortness of breath. Those results prove the reduction in mortality observed in patients receiving CP treatment. This analysis was in accordance with a recent report [40]. In terms of days to hospital discharge and rate of removal from the ventilator, a study evaluating the safety of convalescent plasma therapy based on acute coronavirus, influenza, and Ebola virus infections found no benefit. This corresponds to the findings of a similar study [41].

Compared with other published literature on CP therapy for COVID-19, this meta-analysis has the advantage of involving the most randomized controlled trials. The 13 included articles were all randomized controlled trials of high quality, which did not selectively report the results, and had the most comprehensive outcome indicators. However, we admit that our research has several limitations. First, those included studies differ in size, risk of bias, and external validity. Second, given the limitations of database searches and manual retrieval, it is not certain that all published reports on CP treatment for COVID-19 have been included. Third, the differences between mild, moderate, severe, and critically ill patients were not evaluated, rendering it unclear whether the curative efficacy of CP therapy varied between different populations. Fourth, the follow-up period in all the included publications was insufficient to observe long-term consequences. We will continue to monitor and update the literature analysis as new evidence emerges.

## 5. Conclusions

The safety and potential efficacy of convalescent plasma therapy offer a promising treatment strategy for COVID-19. With no adverse effects, CP treatment can reduce mortality and improve breath and inflammatory cytokines IL-6 and Ferritin in COVID-19. It has little effect on improving virology indicators. As a result, additional high-quality clinical trials are required to validate these results.

## Figures and Tables

**Figure 1:** Flow diagram of database searches and article selection.

**Figure 2:** Risk of bias graph.

**Figure 3:** Risk of bias summary.

**Figure 4:** Sensitivity analysis-mortality.

**Figure 5:** Forest plot-mortality.

**Figure 6:** Sensitivity analysis of the rate of improvement of shortness of breath.

**Figure 7:** Forest plot for the rate of improvement of shortness of breath.

**Figure 8:** Forest plot of the rate of taking off the ventilator.

**Figure 9:** Forest plot demonstrating the improvement of imaging results.

**Figure 10:** Sensitivity analysis for CRP.

**Figure 11:** Forest plot for CRP.

**Figure 12:** Sensitivity analysis of ferritin.

**Figure 13:** Forest plot for ferritin.

**Figure 14:** Forest plot for levels of IL-6.

**Figure 15:** Forest plot for lymphocyte concentration levels.

**Figure 16:** Forest plot for D-dimer.

**Figure 17:** Sensitivity analysis for the incidence of adverse reactions.

**Figure 18:** Forest plot for the incidence of adverse reactions.

**Figure 19:** Sensitivity analysis for days to hospital discharge.

**Figure 20:** Forest plot for days to hospital discharge.

**Figure 21:** Sensitivity analysis for the viral nucleic acid negative conversion rate.

**Figure 22:** Forest plot of viral nucleic acid negative conversion rate and neutralizing antibody-positive conversion rate.

**Figure 23:** Publication bias: (a) mortality; (b) the rate of improvement of shortness of breath.

**Table 1:** Characteristics of the included randomized controlled trials.

No.	Author	Country	The publishing year	Design	Sample size (T/C)	Patients enrolled condition	Treatment group	Control group	CP dose	Outcomes
1	Salman and Mohamed	Egypt	2020	Randomized controlled trial, double-blinded	30 (15/15)	Severe	CP + control group	Supplemental oxygen, noninvasive and invasive ventilation, antibiotic medication, inotrope drugs, renal-replacement therapy, anticoagulants, glucocorticoids, intravenous fluids, interferon, and extracorporeal membrane oxygenation (ECMO)	250 ml/once, one dose	2, 3, 5

2	Ali et al.	Pakistan	2021	Randomized controlled trial, single-blinded	50 (40/10)	Severe and critical	C-IVIG + control group	Airway support, anti-viral medication, antibiotics, fluid resuscitation, hemodynamic support, steroids, painkillers, and antipyretics	0.15, 0.20, 0.25, 0.30 g/kg	1, 2, 3, 4

3	AlQahtani et al.	Bahrain	2021	Randomized controlled trial, open-label	40 (20/20)	Severe and life-threatening	CP + control group	Control of fever (paracetamol) and possible therapy, including anti-viral medications, tocilizumab, and antibacterial medication	200 ml/once, two dose	1, 2, 3, 4

4	Bennett-Guerrero et al.	USA	2021	Randomized controlled trial, double-blind	74 (59/15)	Severe	CP	Standard plasma	240 ml/once, two dose	1, 2, 3

5	Gharbharan et al.	The Netherlands	2021	Randomized controlled trial, open-label	86 (43/43)	Moderate, severe, or life-threatening	CP	Standard of care (not specifically described)	300 ml/once, two dose	1, 2, 3, 5

6	Peter et al.	UK	2021	Randomized controlled trial, open-label	11558 (5795/5763	No data reported	CP + control group	Usual care (not specifically described)	Two units (275 mls ± 155 + 75 mls), two-dose	1, 2, 3

7	Li et al.	China	2020	Randomized controlled trial, open-label	103 (52/51)	Severe and life-threatening	CP + control group	Anti-viral medications, antibacterial medications, steroids, human immunoglobulin, Chinese herbal medicines, and other medications	4–13 ml/kg	1, 2, 3, 5

8	Libster et al.	Argentina	2021	Randomized controlled trial, double-blind	160 (80/80)	Mild	CP	Placebo (0.9% normal saline)	250 ml/once, one dose	1, 3

9	Pouladzadeh et al.	Iran	2021	Randomized controlled trial, single-blind	62 (31/31)	Severe	CP + control group	Chloroquine phosphate, lopinavir/ritonavir, etc	500 ml/once, the second the unit was prescribed if no improvement was observed after 24 h	1, 2, 3, 4

10	O'Donnell et al.	USA, Brazil	2021	Randomized controlled trial, double-blind	223 (150/73)	Severe and critical	CP	Normal control plasma	200–250 ml/once, one dose	1, 2, 3, 4

11	Simonovich et al.	Argentina	2020	Randomized controlled trial, double-blind	333 (228/105)	Severe	CP	Placebo (normal saline solution)	500 ml/once, one dose	1, 2, 3

12	Agarwal et al.	India	2020	Randomized controlled trial, open-label	464 (235/229)	Moderate	CP + control group	Anti-virals (hydroxychloroquine, remdesivir, lopinavir/ritonavir, oseltamivir), broad-spectrum antibiotics, immunomodulators (steroids, tocilizumab), and supportive management	200 ml/once, two-dose	1, 2, 3, 4, 5

13	Rasheed et al.	Iraq	2020	Randomized controlled trial, open-label	49 (21/28)	Critical	CP + control group	Hydroxychloroquine 200 mg twice per day for at least 10 days + azithromycin once 500 mg/day loading dose, followed by 250 mg once per day for 5 days + oxygen therapy + methylprednisolone 40 mg per day	400 ml/once, one dose	1, 2, 3, 5

T: treatment group. C: control group. CP: convalescence plasma. C-IVIG: hyperimmune anti-COVID-19 intravenous immunoglobulin. Outcome: (1) mortality rate; (2) clinical improvement rate; (3) the incidence of adverse reactions; (4) days to hospital discharge; (5) the improvement rate of virology indicators.

## Data Availability

All data generated or analyzed during this study are included in this article.
